# Epidemiological Survey of Thyroid Nodules in 2098 Patients for Routine Physical Examination in Fujian, China

**DOI:** 10.1155/2022/2913405

**Published:** 2022-06-13

**Authors:** Xishun Huang, Yaohui Qiu, Yihui Chen, Lin Chen, Jiao Yi, Xiaohua Luo

**Affiliations:** ^1^Department of Health Medicine, The Affiliated Dongnan Hospital of Xiamen University, School of Medicine, Xiamen University, Zhangzhou, Fujian 363000, China; ^2^Department of Oncology, The Affiliated Dongnan Hospital of Xiamen University, School of Medicine, Xiamen University, Zhangzhou, Fujian 363000, China

## Abstract

**Objective:**

The aim of this study is to establish the prevalence, ultrasound manifestations, and signs of thyroid nodules (thyroid nodules, TNS) in the healthy population, in order to provide a basis for the early diagnosis, treatment, and health education for clinical prevention of thyroid diseases.

**Methods:**

The data of 2098 physical examination clients who underwent thyroid color Doppler ultrasound examination at our hospital's physical examination center from January 1, 2017, to December 31, 2018, were randomly selected, and the prevalence, size, nature, number, and Thyroid Imaging Reporting and Data System (TI-RADS) classification of the thyroid nodules were statistically analyzed.

**Results:**

Of the 2098 results analyzed, 992 cases (47.28%) had thyroid nodules; 327 (15.59%) males and 665 (31.70%) females. The prevalence among females was significantly higher than that among males (*p* < 0.01), and the prevalence increased with age (*p* < 0.05). The composition ratios of multiple nodules and single nodules in each age group were compared, and the difference was statistically significant (*p* < 0.05). Detected thyroid nodules were mainly solid, and they were significantly different compared to the cystic and mixed nodules (*p* < 0.01). The actual classification in our study is consistent with the theory of TI-RADS1∼5 classification.

**Conclusion:**

In conclusion, to sum up, thyroid color Doppler ultrasonography is very important for screening thyroid nodules in healthy people during routine physical examination, especially in high-pressure and high-intensity working environment, post-menopausal women, and men with family members with a history of thyroid cancer. Therefore, high-risk groups are encouraged to have regular thyroid ultrasonography, while health care workers are encouraged to publicize the risk factors of thyroid nodules and the importance of routine thyroid ultrasound examination.

## 1. Background

Today, changes in people's diet structure and the fast-paced nature of work with high pressure have led to a yearly increase in the prevalence of thyroid nodules [1]. Clinically, most thyroid nodules are benign, with only a few that are malignant. Studies show that malignant thyroid nodules account for about 5%–15% of all thyroid nodules [2]. The incidence of thyroid nodules is much higher among middle-agedwomen in whom benign multiple nodules are muchmore frequent than single nodules, while malignant single nodules are much more frequent than multiple nodules [3].

Features of color Doppler ultrasound include on-invasiveness, convenience, and high repeatability and can be used to rapidly acquire the radiographic features within the thyroid lesions. Ultrasonography has become the preferred imaging method for preoperative diagnosis, postoperative follow-up, and screening of thyroid nodules. The improved TI-RADS, when combined with CEUS, could significantly improve the diagnostic accuracy for thyroid nodules, especially for TI-RADS class-4 thyroid nodules. With the increasing popularity of color Doppler ultrasound in routine physical examination, the detection rate of thyroid nodules continues to increase. In order to understand the epidemiological features of thyroid nodules and set a basis for its early diagnosis and prevention, 2098 results of color Doppler ultrasound scans conducted between January 1, 2017, and December 31, 2018, at the physical examination center of our hospital were randomly selected and statistically analyzed. Their epidemiological characteristics and key associations have been summarized and reported as in this paper.

## 2. Materials and Methods

### 2.1. Survey Subjects

From January 1, 2017, to December 31, 2018, a total of 2111 patients were randomly selected for high resolution B-type thyroid ultrasound examination at the physical examination center of our hospital. 13 patients who had previous history of thyroid disease and surgery were excluded, leaving a total of 2098 eligible for the study: 891 males and 1267 females. They had a mean age of 44.02 ± 6.02 years, ranging from 18 to 76 years.  Table 1.

### 2.2. Methods

#### 2.2.1. Philips Color Doppler Ultrasound Machine

Philips color Doppler ultrasound machine was used with the probe frequency adjusted to between 4 and 12 MHz. The patient was positioned in a supine position, the neck assisted with a pillow, and the head tilted back as far as possible to fully expose the thyroid gland. Multiple sections of the thyroid were then scanned, and the size, shape, and number of nodules (one nodule was called a single nodule, and two or more nodes were called multiple nodules), internal echo (the echo formed by ultrasonic rebound by thyroid tissue is divided into low, high, and mixed echo), edge condition, whether there is calcification in the nodule (if there is calcification, it is divided into microcalcification ≤ 1 mm and coarse calcification > 1 mm), aspect ratio, etc. were recorded. The signs of thyroid nodules in different patients were analyzed [4]. Cystic nodules showed low echo, solid nodules showed high echo, and cystic and solid nodules showed mixed echo.

#### 2.2.2. TI-RADS Classification Standard

According to Horvath et al. [5] (Figure 1), the criteria for evaluating malignant thyroid nodules involve the following five key ultrasonic signs: extremely low echo or low echo, solid nodules, fuzzy nodules, fine gravel calcification, and aspect ratio greater than 1. The thyroid nodule is thus classified into TI-RADS (thyroid imaging reporting and data system): TI-RADS category 1: normal gland; TI-RADS category 2: benign nodules, 0% malignant; TI-RADS category 3: possibly benign nodules and malignant nodules <2%; TI-RADS category 4A: there is 1 sign of malignancy, and the probability of malignancy is 5%–10%; TI-RADS category 4b: two signs of malignancy, with a probability of malignancy of 10% to 80%; TI-RADS category 4C: 3 or 4 signs of malignancy and probability of malignancy >80%; TI-RADS category 5: there are 5 malignant signs, and the probability of malignancy is >90%.

### 2.3. Statistical Analysis

Statistical data analysis was conducted using SPSS software, version 21.0. The rate of detection of the thyroid nodules was determined by gender and 6 age groups. The chi-square test (*χ*2) was used to compare the composition ratio of multiple nodules and single nodules in all age groups, with the statistical significance set at *P* < 0.05. Pathological results were taken as the gold standard, and the percentage of malignancy was calculated according to the TI-RADS classification.

## 3. Results

### 3.1. Relationship between the Detection Rate of Thyroid Nodules with Gender and Age

Of the 2098 survey cases, color Doppler ultrasound detected 992 thyroid nodules, with a detection rate of 47.28%. Analyzed by gender, the detection rate was 15.59% in males and 31.70% in females, respectively; the difference between the two is statistically significant (*X*^2^ = 18.306, *P*=0.004).

Stratified by age groups, the detection rate among cases in the 18–29 age group was the lowest and gradually increased with age. Among males, the 60–69 age group had the highest rate (65.38%), while for females, the 50–59 age group had the highest rate (76.51%) (see Table 1, Figures 2 and 3). The detection rate of thyroid nodules in all age groups was statistically significant (*X*^2^ = 57.126, *P*=0.0009).

### 3.2. Relationship between Age, Echo Nature, and the Number of Thyroid Nodules

Of the 992 cases with thyroid nodules, 486 (48.99%) had multiple nodules, while 506 (51.01%) had single nodules. There was significant difference in the constituent ratio of multiple nodules and single nodules at different age groups (*X*^2^ = 8.004, *P*=0.041), and the detection rate gradually increased with increase in age. The composition of the thyroid nodules were mainly solid nodules, which were significantly different from cystic nodules and mixed nodules (*X*^2^ = 24.084, *P* < 0.01) (see Table 2).

### 3.3. TI-RADS Classification of the Nodules

Of the 992 cases with thyroid nodules, 425 cases had TI-RADS class 1 and class 2 (all benign); 336 cases had TI-RADS class 3 (334 benign and 2 malignant); 107 cases had TI-RADS class 4a (102 benign and 5 malignant); 91 cases had TI-RADS class 4B (82 benign and 9 malignant); 24 cases had TI-RADS class 4C (6 benign and 18 malignant); and 9 cases had TI-RADS class 5 (1benign and 8 malignant). The actual malignant percentages of TI-RADS class 1 ∼ 5 were 0, 0, 0.6%, 4.67%, 9.89%, 75.00%, and 88.89%, respectively. See Table 3.

## 4. Discussion

The thyroid is an important endocrine organ of human body. Its main function is to regulate human metabolism, psychological development, physical development, and emotional state. Thyroid nodule (TNs) is a frequently occurring disease in the endocrine system. It is a mass in the thyroid tissue caused by abnormal hyperplasia of thyroid glands for various reasons. The prevalence of thyroid nodules in China continues to increase and is attributed to factors such as population aging, great social pressure, emotional internal injury, autoimmune disease, salt iodization, and living environment [6]; because there are no obvious clinical symptoms in the early stage and the medical history is long, the probability of finding nodules by palpation of thyroid by the first doctor is 3%–7%, and the probability of finding nodules by high-frequency color ultrasound is 20%–76%; at present, most thyroid nodules are usually found accidently in physical examination. When a few patients have signs and symptoms such as pharyngeal discomfort and thick induration of the neck, their disease has developed to the middle and late stage [7]. Clinical research shows that [8], under the high-frequency color Doppler ultrasound probe, it can clearly display the size and number of thyroid nodules with *D* ≥ 0.5 mm and can find thyroid nodules very early, which is of great significance to provide treatment basis for clinicians.

This study discovered that the detection rate of thyroid nodules in randomly selected patients is significantly higher among women (31.70%) compared to men (15.59%), both as a whole (*P* < 0.01) and when stratified by age groups (*P* < 0.01). This result is consistent with a similar study by Luo Jingmei [9]. In our age strata, the women group with the highest detection rate was 50∼59 years old, which was much lower than that of men (60∼69 years old). It can thus be concluded that women generally have a higher incidence of thyroid nodules that gradually increases with increase in age. This could be attributed to female endocrine dysfunction that comes with aging such as those caused by menopause, abuse of health care products, and greater emotional fluctuation in women. So, health care workers should pay more attention to the thyroid ultrasound examination of women during routine physical exam, especially those in the older age category [10]. Though the incidence is much lower in men compared to that in women, studies show that once a nodule is detected in men, especially those with a family history of thyroid cancer, keen attention should be paid to them; serological and cytology examination should be promptly conducted to confirm their nature [11].

Analyzing by types and composition, our results showed that out of the 992 cases with thyroid nodules, 506 (51.01%) had multiple nodules, while 486 (48.99%) had single nodules. There was indeed a significant difference in the composition ratio of multiple and single nodules at different age groups (*X*^2^ = 8.004, *P*=0.041), and the proportion of multiple nodules increased with age. In both genders, the nodules were mainly solid (75.60%), which was statistically different from cystic nodules and mixed nodules (*P* < 0.01). This finding is consistent with the results of two similar studies by Xing et al. [12] and Xu et al. [13]. However, the severity of a thyroid nodule is not necessarily related to its size or number; it is mainly based on its imaging manifestations, such as clear nodular boundaries, integrity of the capsule, nature of internal echo, and level of calcification. Of course, despite these imaging manifestations, the final diagnosis is still arrived at with the help of blood examination results, radionuclide scans, puncture biopsy, etc.

High frequency color Doppler ultrasound is currently the first choice for detecting thyroid nodules [14]. It can accurately determine the size, number, echo nature, and boundary of thyroid nodules. When combined with the TI-RADS classification standard, it can predict preliminary possibilities of benign and malignant thyroid nodules, and in the process, it can provide an objective basis for clinical management of the nodules. According to Kwak et al. [15], who combined ultrasonic signs with pathological biopsy results, they established a TI-RADS classification system that divided thyroid nodules into 5 TI-RADS categories. In our study, the actual malignant percentages according to TI-RADS 1∼5 were 0, 0, 0.6%, 4.67%, 9.89%, 75.00%, and 88.89.0%, respectively, highly consistent with the theoretical malignant percentages of 0, 0, 0.3%∼2.0%, 3.6%∼12.7%, 6.8%∼37.8%, 21.0%∼91.9%, and 88.7%∼97.9% in the Horvath's study. This result in our study is also consistent with another similar study [16]. The TI-RADS classification as proposed by Kwak et al. [15] and Horvath et al. [5] is thus a simple and easy way to operate the tool that has enormous clinical significance in ultrasonic examination of thyroid nodular diseases.

In conclusion, color Doppler ultrasonography of the thyroid has become the first-choice method for routine physical examination of the thyroid, aiding early diagnosis of thyroid diseases. It is advantageous because the whole process is noninvasive, dynamic, and real-time and has great reproducibility [17]. Women are generally more likely to develop thyroid nodules compared to men, and the incidence increases with increase in age, the critical age group being 50–59 years. Therefore, a routine thyroid ultrasound scan, at least every half a year, is encouraged for the high-risk population such as people in a high-pressure and high-intensity working environment, postmenopausal women, and men with a family history of thyroid cancer. As a public health measure, health care workers should continuously educate the population about the risks of developing thyroid nodules and the benefits of regular ultrasound examination in the high-risk group.

## Figures and Tables

**Figure 1:** TI-RADS classification criteria in the present study.

**Figure 2:** The etection rate in males of all ages (%).

**Figure 3:** The etection rate in females of all ages (%).

**Table 1:** Relationship between the detection rate of thyroid nodules with age and gender.

Age (years)	Detection rate % (*n*/*n*)	Males		Females	
		Cases (*n*)	Detection rate (%)	Cases (*n*)	Detection rate (%)
18 ∼ 29	28.48 (137/481)	202	45 (21.74)	274	92 (33.58)
30 ∼ 39	42.82 (185/432)	157	58 (36.94)	275	127 (46.18)
40 ∼ 49	49.56 (227/458)	187	76 (40.64)	271	151 (55.72)
50 ∼ 59	62.12 (182/293)	144	68 (47.22)	149	114 (76.51)
60 ∼ 69	63.86 (159/249)	78	51 (65.38)	171	108 (63.16)
70∼	55.14 (102/185)	58	29 (50.00)	127	73 (57.48)
Total	47.28 (992/2098)	831	327 (39.35)	1267	278 (52.49)

**Table 2:** Comparison of the number and nature of thyroid nodules at different ages (*n* (%)).

Age groups (years)	Cases (*n*)	Number of nodules (%)		Nature of nodules (%)		
		Single	Multiple	Cystic	Solid	Mixed
18∼29	137	91 (66.42)	46 (33.58)	28 (20.44)	96 (70.07)	13 (9.49)
30∼39	185	111 (60.00)	74 (40.00)	36 (19.46)	128 (69.19)	21 (11.35)
40∼49	227	131 (57.71)	96 (42.29)	40 (17.62)	172 (75.77)	15 (6.61)
50∼59	182	75 (41.21)	107 (58.79)	20 (10.99)	148 (81.32)	14 (7.69)
60∼69	159	61 (38.36)	98 (61.64)	17 (10.69)	125 (78.62)	17 (10.69)
70∼	102	37 (36.27)	65 (63.73)	5 (4.90)	81 (79.41)	16 (15.69)
Total	992	506 (51.01)	486 (48.99)	146 (14.83)	750 (75.60)	96 (20.44)

**Table 3:** Relationship between the TI-RADS classification and pathological results of the 992 cases of thyroid nodules.

TI-RADS classification	Cases (*n*)	Pathological (*n*)		Malignant percentage	Malignant percentage
		Cases (*n*)	Detection rate (%)	This study	Horvath's study
Category 1	197	197	0	0	0
Category 2	228	228	0	0	0
Category 3	336	334	2	0.6	0.3∼2.0
Category 4a	107	102	5	4.67	3.6∼12.7
Category 4b	91	82	9	9.89	6.8∼37.8.
Category 4c	24	6	18	75.00	21.0∼91.9
Category 5	9	1	8	88.89	88.7∼97.9

## Data Availability

The datasets used and analyzed during the current study are available from the corresponding author upon reasonable request.
